This article has been retracted.

# Efficacy of using adipose-derived stem cells and PRP on regeneration of 40 -mm long sciatic nerve defect bridged by polyglycolic-polypropylene mesh in canine model

**DOI:** 10.1186/s13287-024-03796-z

**Published:** 2024-07-18

**Authors:** Mona M. Khaled, Asmaa M. Ibrahium, Ahmed I. Abdelgalil, Mohamed A. El-Saied, Aya M. Yassin, Nagy Abouquerin, Hamdy Rizk, Samah H. El-Bably

**Affiliations:** 1 Department of Anatomy & Embryology, Faculty of Veterinary Medicine, Cairo University, Giza, Egypt; 2 Department of Surgery, Anesthesiology and Radiology, Faculty of Veterinary Medicine, Cairo University, Giza, Egypt; 3 Department of Pathology, Faculty of Veterinary of Veterinary Medicine, Cairo University, Giza, Egypt; 4 Department of Biochemistry and Molecular Biology, Faculty of Veterinary Medicine, Cairo University, Giza, Egypt; 5 Department of Physiology, Faculty of medicine, Ain shams University, Cairo, Egypt

**Keywords:** Sciatic nerve regeneration, Neural tube, PRP, Adipose-derived stem cells, Dogs, Growth factors

## Abstract

**Background:**

Sciatic nerve repair becomes a focus of research in neurological aspect to restore the normal physical ability of the animal to stand and walk. Tissue engineered nerve grafts (TENGs) provide a promising alternative therapy for regeneration of large gap defects. The present study investigates the regenerative capacity of PRP, ADSCs, and PRP mixed ADSCs on a long sciatic nerve defect (40-mm) bridged by a polyglycolic polypropylene (PGA-PRL) mesh which acts as a neural scaffold.

**Materials and methods:**

The study was conducted on 12 adult male mongrel dogs that were randomly divided into 4 groups: Group I (scaffold group); where the sciatic defect was bridged by a (PGA-PRL) mesh only while the mesh was injected with ADSCs in Group II (ADSCs group), PRP in Group III (PRP group). Mixture of PRP and ADSCs was allocated in Group IV (PRP + ADSCs group). Monthly, all animals were monitored for improvement in their gait and a numerical lameness score was recorded for all groups. 6 months-post surgery, the structural and functional recovery of sciatic nerve was evaluated electrophysiologically, and on the level of gene expression, and both sciatic nerve and the gastrocnemius muscle were evaluated morphometrically, histopathologically.

**Results:**

Numerical lameness score showed improvement in the motor activities of both Group II and Group III followed by Group IV and the scaffold group showed mild improvement even after 6 months. Histopathologically, all treated groups showed axonal sprouting and numerous regenerated fascicles with obvious angiogenesis in proximal cut, and distal portion where Group IV exhibited a significant remyelination with the MCOOL technique. The regenerative ratio of gastrocnemius muscle was 23.81%, 56.68%, 52.06% and 40.69% for Group I, II, III and IV; respectively. The expression of NGF showed significant up regulation in the proximal portion for both Group III and Group IV (*P* ≤ 0.0001) while Group II showed no significant difference. PDGF-A, and VEGF expressions were up-regulated in Group II, III, and IV whereas Group I showed significant down-regulation for NGF, PDGF-A, and VEGF (*P* ≤ 0.0001).

**Conclusion:**

ADSCs have a great role in restoring the damaged nerve fibers by secreting several types of growth factors like NGF that have a proliferative effect on Schwann cells and their migration. In addition, PRP therapy potentiates the effect of ADSCs by synthesis another growth factors such as PDGF-A, VEGF, NGF for better healing of large sciatic gap defects.

## Introduction

Sciatic nerve injury is the most prevalent syndrome occurring in the peripheral neuropathy regarded to hindlimb nerves [1]. It commonly occurs as a result of trauma, falls, compression by a cyst, tumors, or bone fracture and characterizes by muscle atrophy, knuckling, and animal’s inability to bear weight on its limbs [2]. The peripheral nerves have a limited regenerative capacity, particularly in large-sized defects depending on the severity and the extent of injury [3]. Peripheral nerves can regenerate in minor injuries including neuropraxia and/or axonotmesis, while in severe injuries as neurotmesis the nerve loses its ability to regenerate, and a painful neuroma or fibrous tissue is developed [4, 5].

Among a wide variety of alternative strategies for nerve regeneration, tissue-engineered nerve grafts (TENGs) have been developed as a promising therapy for Peripheral Nerve Injury (PNI) and primarily consist of a neural scaffold loaded with supporting cells and/or growth factors [6]. Nerve tubularization with a synthetic conduit like poly-glycolic-acid mesh (PGA) enhances growth of nerve cells by bridging the gap between the proximal and distal nerve stumps and preventing the haphazard growth pattern and irregular innervation [7].

Mesenchymal stem cells (MSCs) are pluripotent adult cells that recently grown to be a highly attractive source of cell implantation for tissue engineering due to their capacity for self-renewal, rapid proliferation, and multilineage differentiation [1, 8]. Adipose-derived stem cells (ADSCs) are considered an accessible kind of adult stem cell that has become the focus of research for neuronal regeneration. They can be differentiated into various types of cells such as chondrocyte, adipocyte, myocyte, osteocyte, and neurons. They possess unique characters such as they are more easily harvested from any fat rich sources, low immunogenicity, faster proliferation, high cellular density, and the ability to be collected in large quantities with minimal invasive techniques [1, 8–11].

Recently, Platelet-rich plasma (PRP) is considered a rich source of many neurotrophic factors that enhance the repairing capacity of nervous tissue. Moreover, it has been proved that PRP afford a neuroprotection against cell apoptosis, trigger angiogenesis, stimulate axonal regeneration, and decrease the inflammatory response for optimal neuronal growth [12–14]. So, the aim of the present study was to investigate the regenerative capacity of PRP, adipose derived stem cells (ADSCs) and PRP mixed ADSCs on a long sciatic nerve defect (40-mm) bridged by a polyglycolic polypropylene (PGA-PRL) mesh in experimental dog model. Clinical, electrophysiological, histopathological, biochemical and morphometrical parameters were used for evaluation of neural growth and axonal remyelination.

## Material and method

### Ethical approval

All study procedures were approved by the Institutional Animal Care and Use Committee (IACUC) at the Faculty of Veterinary Medicine, Cairo University, Egypt; with number (Vet CU 01122022595). The study was carried out in compliance with the ARRIVE guidelines.

### Animals

The study was conducted on 12 apparently healthy adult male Mongrel dogs with average weight (15–20 kg) and age (1–3 years). Animals were housed in individual cages at the Department of Surgery, Radiology and Anesthesiology, Faculty of Veterinary medicine, Cairo University. The inclusion criteria included normal response to neurological examination of both fore and hind limbs. All animals were allowed 2 weeks for acclimatization before surgical operations. During the period of acclimatization, animals were treated by deworming tablets (prazitab®, O.L.KAR.) with dose of one tablet for 10 Kg Bwt. Animals were fed twice time daily using commercially produced dog pelleted food and offered fresh drinking water *ad-lib.*

### Experimental design

After the end of the acclimatization period, animals were randomly divided into four equal groups (*n* = 3 in each group) where the right hind limb received the different treatments according to their group while the left hind limb represented as control negative. In Group I, only the neural tube was sutured between the two nerve stumps (scaffold group) represented as positive control, ADSCs group (Group II), PRP group (Group III) and ADSCs + PRP group (Group IV). The end of the experiment was 6 months post treatment.

### Experimental procedures

#### Adipose-derived stem cells (ADSCs) preparation and characterization:

##### Isolation of stromal vascular fraction (SVF)

Under general anesthesia, a small skin incision was applied at Linea-alba just caudal to xiphoid cartilage and after exposure of the peritoneum, about 15 g of fat adherent to the parietal peritoneum was collected (Tela subserosa or peritoneal fat). Under a complete sterile laminar air flow, the fat was washed with PBS to remove excess blood and debris and then minced into small pieces using surgical blades until a fat emulsion is formed. Then, the emulsion was treated with equal volume of 0.075% collagenase type II (Sigma-Aldrich, St. Louis, MO, USA) for 60 min at 37 °C and a 5% CO2 incubator with continuous agitation in a rotatory wheel. After that, an equal volume of Dulbecco’s Modified Eagle’s Medium (DMEM) containing 10% fetal bovine serum (FBS) was added to neutralize the enzyme activity. The mixture of cells, collagenase, and media was centrifuged at 2000 rpm for 10 min. for pelleting of cells and removing the cellular debris in supernatant. The pelleting was repeated three times with PBS at 2000 rpm for 10 min. at the last round of centrifugation, the pellet was dissolved in 1 ml of DMEM and mixed with 1 ml of sodium alginate.

##### Culturing and expansion of ADSCs

In a sterile culture flask (75-cm^2^) containing DMEM high glucose with 10% FBS and 100 mg/mL penicillin/streptomycin, ADSCs were incubated at 37 °C with 5% humid CO2. After 48 h, the medium was replaced for removal of non-adherent cells and the adherent was supplied by complete medium and cultured for 7–12 days until a cell confluence of 80-90% was achieved regarding to the first passage (P1) cells. During this period the culture media was changed every 3 days until reaching the third passage.

#### ADCSs characterization

The cells of passage three were harvested by trypsinization process using a trypsin EDTA solution for 5 min in the incubator, followed by PBS washing to remove excess trypsin. The cell pellet was then incubated for one hour with 1% bovine serum albumin containing primary antibodies against the following cell surface markers: CD 34, CD73, CD45, CD44, CD90 and CD105. The cells were then incubated for 30 min with the secondary antibody before immunophenotyping using a fluorescence activated cell sorting cell analyzer (CytoFLEX, Beckman Coulter, United States).

#### ADSCs differentiation

The Mesenchymal phenotyping capacity of ADSCs was demonstrated by incubating cells of passage three into three different media: adipogenic, osteogenic, and chondrogenic. The cells were trypsinized, loaded on 6-well plates at a density of 20 × 10^3^cells/cm2 and differentiated invitro using adipogenesis kits (A1007001; Gibco StemPro, USA) or osteogenesis kits (A1007201; Gibco StemPro) or Chondrogenesis Kit (A1007101; Gibco StemPro) for 3 weeks. The corresponding media was changed every 3 days. A 0.5% Oil Red O (marker for intra-cellular lipid accumulation), Alizarin Red S (marker for extra-cellular matrix calcification), and Safranin O (trigger of chondrocyte development) stains were used for staining of cells differentiated from the adipogenic, osteogenic, and chondrogenic media respectively.

#### Preparation of autologous PRP

Autologous PRP was collected and prepared according to the previously described method by [15]. Briefly, the blood samples were collected aseptically via jugular vein on an anticoagulant citrate dextrose solution (1:9) under the effect of xylazine 2% (1 mg/kg) as a tranquilizer. A double centrifugation cycles were applied. The first cycle achieved 3000 rpm for 3 min and the plasma in the supernatant was collected in another new tube that entered the second cycle at 4000 rpm for 15 min. After the second centrifugation cycle, PRP was formed at the lower third of the tube and gathered to be mixed with 5 ml sodium alginate in a sterile petri-dish and then collected in a needle with nozzle to be injected directly into the mesh.

### Preparation of neural tube

Commercially available poly-glycolic acid poly-propylene mesh (prosorb mesh® formerly sutures India Pvt.Ltd.) was cut into 4 cm width and 5 cm length then it warped manually and sutured using 4 − 0 vicryl to mimic the neural tube (1.5 cm diameter and 5 cm length). The warped mesh was autoclaved before operation **(**Fig. 1).

#### Anesthesia

The dogs were premedicated by intramuscular injection of atropine sulfate® (Atropine sulfate®1 mg/ml Med.Co., A.R.E) with dose of 0.05 mg/kg and xylaject 2%® (Xyla-Ject® 2% ADWIA Co., A.R.E.) with dose of 1 mg/kg. General anesthesia was induced by I/V injection of ketamine® (Ketamar® 5%, Amoun Co. A.R.E) with dose of (10 mg/kg) and maintained by I/V injection of pharcopental® _(_Thiopental®, EPICO, A.R.E) with dose of 25 mg/kg.

#### Surgical procedures

Under general anesthesia, 5 cm surgical incision was applied in the right thigh region just distal to the ischial tuberosity (major landmark) and extended between the biceps femoris and semitendinosus muscle then, blunt dissection till exposure of the sciatic nerve. Surgical excision of 2 cm segment was done then the prepared neural mesh was sutured to the proximal and the distal stumps of the nerve using 4 − 0 vicryl that resulted in a 40 mm long nerve gap due to the traction of the nerve. In Group I, only the neural tube was sutured between the two nerve stumps while ADSCs, PRP and mixture of PRP and ADSCs on sodium alginate (4 ml) (as a vehicle) was injected in the tube in Group II and III, and IV respectively before suturing of the distal part of the mesh with the distal stump of the nerve. The muscles and subcutaneous tissue were sutured simple continuous pattern using 2 − 0 vicryl and the skin was sutured simple interrupted pattern using 0-nylon sutures **(**Fig. 2**).**

#### Post-surgical care

Post-operative care included analgesic Carprofen100mg (Rimadyl®, Zoetis, A.R.E) with dose of 4.4 mg/kg once daily for 3 days orally and Antibiotics Amoxicillin and clavulanic acid (synolux®, Zoetis, A.R.E) with a dose of 1 ml/20kg once daily for 6 days I/M. Post-operative evaluation included daily monitoring appetite and changes in animal behavior, and monthly evaluation of lameness score.

### Clinical evaluation

#### Numeric lameness scoring system

All animals in each group were monthly examined till the end of the experiment at 6th month to determine the degree of lameness of the affected limb during walking. Grading was taken score from (0–5) where (0) indicates the worst case while (6) indicates sound movement **(**Table 1**).**

**Table 1:** Describe a numerical scale for lameness

Score	Description
Score 0	Paw knuckling and dragging of pelvic limb without any correction even after 10 steps
Score 1	Paw knuckling and dragging of pelvic limb with correction after 8-10 steps then, Paw dragging again
Score 2	Paw knuckling and dragging of pelvic limb with correction after 5-7 steps then, Paw dragging again
Score 3	Paw knuckling and dragging of pelvic limb with correction after 3-4 steps then, Paw dragging again
Score 4	Paw knuckling and dragging of pelvic limb with correction after 1-2 steps then, Paw dragging again
Score 5	Sound movement without Paw knuckling and/or dragging of pelvic limb after 10 steps then, Paw dragging for 2 steps and then sound movement again
Score 6	Sound movement without Paw knuckling and/or dragging of pelvic limb

#### Electrophysiological assessment

The animals were undergoing general anesthesia via I/V injection of ketamine (10 mg/kg) and positioned in a lateral recumbency. The hair was removed, and the skin was cleaned with alcohol. Surface bipolar stimulation was conducted through Trutrace (Czech Republic, Deymed); traveler 4 Chanel system version 7. The surface electrodes were slightly coated with conductive gel (10–20 gel, USA, Weaver and 565 company) and used for measuring the motor nerve conduction parameters of tibial nerve. The active electrode was placed over the most prominent part of gastrocnemius muscle. The motor responses were recorded by applying the supra- stimulus at two sites: a proximal stimulating point just caudal to the greater trochanter and a distal one at the distal third of thigh region. The settings of the device were adjusted involving monitor time at 200 milliseconds (ms), stimulus duration at 0.2 msec, stimulus rate at 1 Hz (Hz), low frequency filter at 20 Hz and high frequency filter at 3 kHz (KHz). Analysis time is 50 ms for motor studies. Also, initial sensitivity was 2 millivolts (mV) for motor nerve conduction and then increased or decreased according to the recorded response. The following measurements were estimated at 1 and 6 months post-surgically: distal latency (DL), duration, amplitude of the CMAPs( Compound muscle action potentials), conduction velocity (CV) and ratio of degeneration [16]. For every measurement, the stimulation was performed five times, and the average values were applied.

Measuring the aforementioned parameters came after supramaximal stimulation was achieved. By progressively raising the simulation current, supra-maximal stimulation is attained. Assuming supramaximal stimulation is achieved, Supra-maximal stimulation reached via gradually increasing the simulation current. The current is slowly increased from a baseline 0 mA, usually by 5–10 mA increments, till a point where the current increase is not associated with increased in the amplitude of CMAPs, assuming that supramaximal stimulation is reached. Then, the stimulating current increased by 20% to ensure the supra maximal stimulation [17]. After reaching Supramaximal stimulation, the above mentioned values were obtained and after 6 month the ration of degeneration were calculated by measuring the percentage of CMAPs amplitude reduction from 1 month.

#### Morphometrical analysis

All dogs were euthanized at the end of the study after 6 months of treatment by thiopental sodium 1gm intravenously. The lateral and medial heads of gastrocnemius muscle were dissected from the lateral and medial heads of supracondylar tuberosity of the femur till the calcaneal tendon in both treated and contralateral limbs. The length, width and weight of each muscle were estimated and documented as a ratio between the operated and the contralateral.

### Histopathological assessment

#### Nerve histology

Sciatic nerve samples from three dogs of each study group were analyzed. Samples were fixed in 10% neutral buffered formalin, dehydrated with alcohol then cleared in xylene, embedded in paraffin wax, and sectioned at 5 μm for routine histopathological examination, morphological, and histochemical analyses. MCOLL histochemical method was achieved for morphological pattern evaluation and quantification of myelin sheath and stromal collagen fibers contents [18]. Nerve regeneration was evaluated at three levels: proximal, middle, and distal stumps of the nerve.

#### Histopathological analysis of the gastrocnemius muscle

Several segments were taken from the mid-belly part of gastrocnemius muscle and preserved in 10% neutral buffered formalin and processed in alcohol, xylene and embedded in paraffin block then sectioned at 5 μm for routine histopathological examination. Masson trichome satin was carried out for determination the degree of fibroplasia. The morphometric quantitative analysis of the muscle fiber cross-sectional area was executed as reported previously [19]. The image analysis was performed for collagen fiber evaluation and quantification on transverse sections of gastrocnemius muscle stained with Masson trichrome stain [7].

### Gene expression analysis

#### Samples collection

A 6-mm piece of sciatic nerve was cut proximally and distally from the point of transection from both the right limb (treatment groups) and the contralateral left limb (control negative). The samples were immediately frozen in -196 °C liquid nitrogen, and stored at -80 °C.

#### Total RNA extraction and cDNA synthesis

Total RNA was isolated using a total RNA purification kit (Jena Bioscience, Germany, Cat. #PP-210 S) according to the manufacturer’s instructions. The RNA concentration and purity were ascertained using Nanodrop ND-1000 Spectrophotometer (Thermo Scientific). The total RNA was then reversely transcribed using the Revert Aid First Strand cDNA Synthesis Kit (Thermo Scientific, USA, Cat. #K1622).

#### Real-time qPCR and gene expression analysis

The primer sequences for the vascular endothelial growth factor (VEGF), platelet-derived growth factor -A (PDGF-A), and nerve growth factor (NGF) genes were designed using Primer 3 software and illustrated in **(**Table 2**).** The mRNA expression level of each gene was determined relative to GAPDH as an endogenous reference gene through a fluorescence-based real-time detection method using iQ SYBR® Green Supermix (Bio-Rad 1,708,880, USA) according to manufacturer instructions. The cycle threshold (Ct) values were obtained using Bio-Rad iCycler thermal cycler and the MyiQ real-time PCR detection system. The cycling protocol was set as follows: 95 °C for 3 min (initial denaturation) and then 40 cycles of denaturation at 95 °C for 15 s, annealing at 60 °C for 30 s, and extending at 72 °C for 30 s. Each assay was performed in triplicates and no-template negative control (NTC) was included; the expression relative to control was calculated using the Eq. 2-ΔΔCT [20].

**Table 2:** Showed Primer sequences for targeted and normalizer genes of Canis lupus familiars

Genes	Forward primer	Reverse primer	Product size	REF./accession No.
GAPDH	5-AGGTCGGAGTCAACGGATTT-3	5-ATCTCGCTCCTGGAAGATGG-3	230	[21]
VEGF	5-TCTGACTAGGAGTTCGGGGA-3	5- CCCTTCCTCCACCAATGTCT-3	214	[21]
PDGF-A	5- CCACCTATGCATCACTTCCTAAA -3	5-TTGGTTCACGCATAGTTCTCTC -3	110	XM_038667633.1
NGF	5-CTGGGAGAGGTGAACATTAACA-3	5-GTAGGAGTTCCAGTGCTTGG-3	123	[22]

### Statistical analysis

Statistical analysis was performed using one-way ANOVA (analysis of variance) to compare the means of the different groups with GraphPad prism 8 software. If there was a significant overall difference between groups, pairwise comparisons were conducted using post hoc Tukey’s multiple comparisons test. Data were presented as the mean ± SD. Values of *P* < 0.05 were considered statistically significant.

## Results

### Stem cell characterization

#### Flow cytometry of isolated cells

Flow cytometric analysis of autologous ADSCs (third passage) for surface markers shown that CD73 (96.04%), CD105 (92.04%), CD9 (90.04%) and CD44 (88.02%) were positively expressed while CD34 (0.16%) and CD45 (0.56%) were negatively expressed which indicating that the isolated cells possess mesenchymal stem cell characteristics as shown in Fig. 3A.

#### Stem cell differentiation

Multi-lineage differentiation power of ADSCs were demonstrated through their positive reaction for Oil Red O, Alizarin Red S and Safranin O stains as shown in Fig. 3B. Adipogenic differentiation was detected by red color of accumulated fat vacuoles by Oil Red O staining while Alizarin Red S detected the mineral deposition within the cell matrix which illustrated the osteogenic capacity. Chondrogenic differentiation was noticed by adding Safranin O that stimulates chondrogenic development.

## Clinical evaluation

### Numeric lameness scoring system

Lameness score of all animals was taken monthly. After 3 months, Group II (ADSCs) showed progressed improvement with weight bearing score 6 in one animal while 2 animals showed score 4 which is the highest group in lameness improvement followed by Group III and Group IV. At the end of the study both Group II and Group III showed the highest improvement in lameness score followed by Group IV. The Group I (scaffold group) showed the least improvement in lameness score with an average score of 2.7 **(**Fig. 4**).**

### Electrophysiological assessment

Regarding to the changes of motor nerve conduction studies, Group I (scaffold group) showed a significant reduction in the amplitude after one and 6 months (0.6 ± 0.06 mV, 1.3 ± 0.45 mV, respectively) in comparison to the contralateral limb (17.3 ± 1.2 mV) with *P* ≤ 0.0001, while Group III (PRP group) showed a significant increase in the axonal function after 6 months (1.96 ± 0.46 mV) compared to one month (1.13 ± 0.15 mV) with *P* ≤ 0.0001. However, there were no significant differences in the conduction velocity of both groups from one months to 6 months. Moreover, Group II (ADSCs group) showed an increase in the conduction velocity after 6 months (45.33 ± 2.60 M/S) in compared to one month (40.33 ± 5.92 M/S) with no statistically significant variation compared to the contralateral limb (63.66 ± 5.78 M/S). In comparison to other treated groups, Group IV (PRP + ADSCs group) showed both axonal and myelin function improvement after 6 months (58.00 ± 4.041 M/S, 2.73 ± 0.27 mV, respectively) in comparison to one month (35.66 ± 8.45 M/S, 2.1 ± 0.86 mV, respectively) with the least ratio of degeneration (83.22 ± 1.64%) than other groups after 6 months **(**Table 3; Fig. 5**).**

**Table 3:** Illustrate the electrophysiological parameters of motor activity of tibial nerve in differient treated group and the ratio of degenration of nerve in compared to the contralateral limb

Parameter	Scaffold	ADSCs	PRP	PRP + ADSCs
**Axonal function**				
Amplitudes (mV)				
Contralateral limb	17.3 ± 1.2	21.5 ± 1.23	27.66 ± 1.24	16.3 ± 0.46
1 month	0.6 ± 0.06	2.36 ± 0.43	1.13 ± 0.15	2.1 ± 0.86
6 months	1.3 ± 0.45	3.33 ± 0.22	1.96 ± 0.46	2.73 ± 0.27
P1	*P* ≤ 0.0001(****)	*P* ≤ 0.0001(****)	*P* ≤ 0.0001(****)	*P* ≤ 0.0001(****)
P2	*P* ≤ 0.0001(****)	*P* ≤ 0.0001(****)	*P* ≤ 0.0001(****)	*P* ≤ 0.0001(****)
P3	ns	ns	*P* ≤ 0.0001(****)	ns
Ratio of degeneration (%)				
Contralateral limb	------	------	------	------
1 month	97.45 ± 0.31	88.89 ± 2.18	93.47 ± 0.37	86.81 ± 5.54
6 months	95.12 ± 1.93	84.49 ± 0.47	88.86 ± 1.9	83.22 ± 1.64
P1				
P2				
P3	ns	ns	ns	ns

Parameter	**Scaffold**	**ADSCs**	**PRP**	**PRP + ADSCs**
**Myelin function**				
Distal latency (DL) (ms)				
Contralateral limb	2.36 ± 0.15	2.2 ± 0.1	2.2 ± 0.057	2.23 ± 0.09
1 month	3.06 ± 0.09	2.43 ± 0.17	4.833 ± 0.44	2.7 ± 0.43
6 months	4.83 ± 0.44	3.13 ±0.15	3.633 ± 0.21	2.4 ± 0.06
P1	ns	ns	*P* ≤ 0.01 (**)	ns
P2	*P* ≤ 0.01 (**)	*P* ≤ 0.01 (**)	*P* ≤ 0.05 (*)	ns
P3	*P* ≤ 0.01(**)	*P* ≤ 0.05 (*)	ns	ns
Conduction velocity (M/S)				
Contralateral limb	73 ± 5.51	63.66 ± 5.78	70.66 ± 2.60	65.67 ± 10.11
1 month	46.66 ± 3.71	40.33 ± 5.92	60 ± 3.46	32.67 ± 6.360
6 months	38 ± 11	45.33 ± 2.60	44 ± 7.5	58.00 ± 4.041
P1	ns	*P* ≤ 0.05 (*)	ns	*P* ≤ 0.05 (*)
P2	*P* ≤ 0.05 (*)	ns	*P* ≤ 0.05 (*)	ns
P3	ns	ns	ns	ns

ms: millisecond, mV: millivolt, M/S: meter per second, P1: contralateral vs. 1 month, P2: contralateral vs. 6 months., and p3: 6 months vs. 1 month

### Morphometrical analysis

The muscles of contralateral limbs serve as a reference value to assess the percentage of muscle atrophy in different groups. All results were calculated as means for all evaluated parameters as shown in **(**Table 4**).** The ratio of gastrocnemius muscle weight was higher in Group II (ADSCs group) (**56.68%)**, Group III (PRP group) **(52.06%)** and Group IV (PRP + ADSCs group )(**40.69%)** in compared to Group I (scaffold group )(**23.81%)** that consider the least group in the muscle weight. There is no significant difference in the ratio of muscle length in all groups. The ratio of muscle width was much better for ADSCs (**78.32%)**, PRP (**70.85%)** and PRP + ADSCs (**67.56%)** groups compared to scaffold group (**56.30%)**.

**Table 4:** Illustrate the ratio of gastrocnemius muscle regeneration in different treated groups

Animal group	Weight (gm)			Length (cm)			Width (cm)		
	Normal	Defected	Ratio	Normal	Defected	Ratio	Normal	Defected	Ratio
Scaffold group	41.9	9.98	**23.81%**	12	12	**100%**	5.66	4.33	**56.30%**
ADSCs group	27.75	15.73	**56.68%**	12	12	**100%**	7.66	6	**78.32%**
PRP group	25.14	13.09	**52.06%**	12	12	**100%**	7	4.96	**70.85%**
PRP + ADSCs	43.45	17.68	**40.69%**	14	13	**92.85%**	6.83	4	**67.56%**

### Histopathological assessment

#### Morphological analysis of the regenerative sciatic nerve

Morphological analysis of the regenerated sciatic nerves was done to observe the three levels: the proximal part to the conduit, middle part of the conduit and distal nerve stump. Examination of the un-injured collateral (control negative) sciatic nerve sections of treated dogs showed normally well-organized and arranged myelinated fibers and Schwann cells. while Group I (scaffold group) displayed marked retardation in nerve regeneration as the proximal part to conduit contained large quantity of fibrous tissue between nerve fibers, as well as the fibrous tissue was increased in the middle portion of the conduit with poor alignment of regenerated fascicles. Wallerian degeneration was markedly seen at the distal portion to the conduit beside high collagen content. In the Group III (PRP group), the proximal part to the conduit mostly had a normal appearance intact myelinated nerve fibers with proliferation of Schwann cells beside abundant blood capillaries. The nerve regeneration process was reached to the middle part of the conduit with prominent axonal sprouting and numerous regenerated fascicles with moderate axonal alignment. Angiogenesis process was seen with minimal interneural scar formation. Also, the regeneration process reached the distal part with obvious Schwann cells proliferation and newly formed blood capillaries. Similarly, Group II (ADSCs group) exhibited the same finding as Group III in proximal and distal part to the conduit, however the middle part of the conduit exhibited more organized regenerated fascicles supported with well-developed blood vessels. On the other hand, Group IV (PRP + ADSCs group) exhibited more regenerative process with highly organized and well-mannered axonal alignment in proximal, middle, and distal parts of the conduit in addition to evident revascularization and Schwann cells proliferation especially in middle and distal parts of the conduits **(**Fig. 6**).**

The MCOLL histochemical staining was confirmed the difference amount of collagen fibre and the regenerated myelin among different parts of experimental groups **(**Fig. 7**).** In Group I (scaffold group), the regeneration process was in a random distributed manner with disorganized nerve fascicles and a high collagen fibre content present in the proximal and middle part of the conduit, to the distal part of the conduits marked demyelinated axon was observed with high collagen fibre content. Despite the treated groups, proximal part to the conduit were considerably had organized well-defined myelin and collagen content. In the Group III (PRP group), the nerve regeneration process attained the middle part of the conduit with regenerated nerve fascicles that also reached the distal part of the conduits. Likewise, the finding in Group II (ADSCs group) as the remyelination was observed at the middle and distal part of the conduit in more organized manner than Group III, however they approximately had the same myelin content with no significant difference between them. Furthermore, a higher significant remyelination was present in Group IV (PRP + ADSCs group) than in the other groups which indicated by the well organized and abundant positive myelin staining regenerated nerve that more prominent in the middle and distal parts of the conduit.

#### Histopathological analysis of the gastrocnemius muscle

Morphometric and morphological analysis of gastrocnemius muscle after 6-month post-surgery revealed normal muscle fiber that uniform in size with peripheral nuclei in uninjured side that considered as control negative group. However, Group I (scaffold group) exhibited marked muscular atrophy, hyperplasia of adipocyte in addition to degeneration, necrosis, and hyalinization of muscle fibers with stromal scirrhous reaction. Noticeable improvements were recorded in treated groups in compared to Group I (scaffold group) as the cross-sectional area of gastrocnemius muscle was significantly inclined in treated groups in comparison to Group I (scaffold group). The cross-sectional area of gastrocnemius muscle of Group IV (PRP + ADSCs group) was markedly elevated in comparison to both Group III (PRP) and Group II (ADSCs) treated groups. There was no statistically significant difference between Group III (PRP) and Group II (ADSCs) groups. Regarding collagen fiber content, it was evaluated and quantificated with Masson trichrome stain. Normal fibrous connective tissue content between muscle fibers and bundles was present in normal group. Contrastingly, the collagen fibers content between muscle fibers and bundles was increased in Group I (scaffold group). However, the collagen content was significantly reduced in the treated groups (Group II, III, and IV) in comparison to scaffold group. As to the treated group, Group IV (PRP + ADSCs) group showed the least collagen content compared to other treated groups, no statistical significance difference detected between either Group III (PRP) and Group II (ADSCs) groups. From the previous parameters, gastrocnemius muscle reinnervation was increasingly enhanced in Group IV (PRP + ADSCs) group then in Group III (PRP) and Group II (ADSCs) groups in the same level **(**Fig. 8**).**

### Gene expression analysis

The present study investigated the expression levels of NGF, PDGF-A, and VEGF for both proximal and distal nerve cuts for the sciatic nerve. NGF expression levels at the proximal nerve cut showed significant up-regulation for both Group III (PRP)and Group IV (PRP + ADSCs) by (1.8, 2) folds; respectively and Group I (scaffold group) showed significant down-regulation to (0.36) fold (*P* ≤ 0.0001), whereas the Group II (ADSCs group) showed no significant difference in comparison to the control negative group **(**Fig. 9A**).** Regarding the distal cut, all the treated groups showed significant down-regulation to (0.27,0.73, 0.55, 0.51) folds for the Group I, II, III, and IV; respectively in comparison to the control negative group with no significant difference between the Group III and Group IV (Fig. 9B**).**

PDGF-A expression levels at the proximal nerve cut showed significant up-regulation for Group II (ADSCs), Group III (PRP), and Group IV (PRP + ADSCs) by (1.2,1.8, 2.8) folds; respectively with superiority for Group IV. Group I (scaffold group) showed significant down-regulation to (0.57) fold (*P* ≤ 0.0001) **(**Fig. 9C**).** The distal cuts of all the treated groups showed significant down-regulation to (0.35, 0.7 ,0.73) folds for the scaffold, ADSCs, and PPR, except for the PRP + ADSCs which showed significant up-regulation by (1.33) fold (*P* ≤ 0.0001); respectively in comparison to the control negative group **(**Fig. 9D**).**

VEGF expression levels at the proximal nerve cut showed significant up-regulation for ADSCs, PRP, and PRP + ADSCs by (1.7, 1.8, 3.7) folds; respectively with superiority for PRP + ADSCs. The scaffold group showed significant down-regulation to (0.37) fold (*P* ≤ 0.0001) **(**Fig. 9E**).** The distal cuts of all the treated groups showed significant down-regulation to (0.3, 0.6, 0.530.45) folds for the scaffold, ADSCs, PPR, and PRP + ADSCs (**P ≤ 0.0001**); respectively in comparison to the control negative group **(**Fig. 9F**).**

## Discussion

Long sciatic nerve defects caused by trauma or after surgical intervention become a major clinical challenge facing surgeons and clinicians as it exceeds the nerve self-repair mechanism after injury. Tissue engineering provides a promising therapy for regeneration of damaged axons when a neural tube alone fails to improve it. Tissue engineered nerve grafts (TENGs) help to regenerate the injured nerve fibers by incorporating several types of supporting cells and/or growth factors in a neural conduit that provide the optimal microenvironment required for nerve regeneration.

Polyglycolic acid (PGA) and polypropylene polymers were used as an artificial neural scaffold in our investigations. PGA polymers have been widely used in combination with other synthetic materials. PGA polymers were used as a neural scaffold in combination with collagen fibers coated in laminin [23], with chitosan [7, 23–27] and with collagen [28] [6]. investigated the effect a chitosan/silk scaffolds for repairing 60-mm sciatic gap in dog.

Introduction of stem cells and/or PRP in the synthetic mesh had a greater restoration of locomotive activities when compared with non-grafted group. These findings were in the same line with [6].

In the present study, a new numerical lameness score (0–6) was used for evaluation of the gait soundness after sciatic injury based on the ability of the affected hind limb to forward movement with or without paw knuckling. Monthly lameness score analysis was recorded. Both ADSCs and PRP groups showed marked and rapid restoration of the locomotor activity. ADSCs mixed PRP showed significant improvement in locomotion activity when compared to the scaffold group [6, 7]. reported that introduction of a neural scaffold mixed with autologous MSCs enhanced the regeneration capacity in a large nerve gas (60 mm) more than scaffold alone.

Electrophysiologically, all treated group exhibited an improved ratio of degeneration after 6 months, while the scaffold group was the least one. These findings explain the regenerative effect of ADSCs and PRP treatment in axonal functional recovery. Furthermore [7], found that there were no significant differences in the CMAP amplitude between autograft and TENG groups (bone marrow stem cells on PGA scaffold) and the parameter in the scaffold group was lower than that in the autograft or TENG group.

In line [29], reported that both the conduction velocity and CMAPs (compound muscle action potential) were significantly higher in MSC (mesenchymal stem cells) injected treated groups than in the ANA (a cellular nerve allograft) group (scaffold ), that result support our finding where, there is an increase in axonal and myelin functions in both ADSCs (Group II) and PRP + ADSCs (Group IV) after 6 months, in comparison to one month.

The CMAPs was higher in Group II (ADSCs) than in Group III (PRP), that was in contrast to [30] in rat, which demonstrated that CMAPs in PRP group was higher than the MSCs group (bone marrow mesenchymal stem cells), moreover both PRP and MSCs were significant higher in comparison to control group [18]. added that the treated collagen conduit seeded with human umbilical cord stem cells (hUC-MSCs) increased the CMAPs after 9 months surgery and the CMAPs amplitude ratio was significantly higher in treated MSCs group compared with the LOCC-alone group (represent scaffold group in our study).

In disagreement with [31] who said that there were no significance difference in the nerve conduction velocity between different grafted groups after five months Although in our work, the conduction velocity was significantly increased in Group II (ADSCs) and Group IV (PRP + ADSCs) after 6 months. In addition, we recorded that myelin function in Group IV (PRP + ADSCs) has no statistical significance variation from the contralateral limb.

Adipose derived-stem cells (ADSCs) are pluri-potent stem cells that can be differentiated into osteocyte, chondrocyte, and neurons. Besides their faster proliferation capacity and easy handling technique, they are highly preferred for transplantation due to their lower immunogenicity and higher immune-compatibility [32]. ADSCs had a potential therapeutic effect in repairing sciatic nerve injury in rats and rabbits [11, 32–37]. PRP had an important therapeutic role in nerve damage as its products function as a neurogenic modulator and a neuroprotective [29, 38]. Although PRP had been used in many studies [1, 29] but its combination with ADSCs was not reported in treatment of sciatic neuropathy in dogs.

In our study, the comparison between measured width and weight between affected and contralateral gastrocnemius muscle was used as indicator of muscle improvement. Ratio of muscle regeneration revealed that both ADSCs and PRP groups showed highest ratio of improvement followed by the ADSCs mixed PRP group. There was no significant variation in the regeneration ratio between the PRP and adipose groups and these findings were correlated with the numerical lameness score results. The later result was in the same line with [18] who concluded that the net weight of gastrocnemius muscle was significant higher in LOCC/hUC-MSCs group (longitudinally oriented collagen conduit/human umbilical cord-mesenchymal stem cells) than in the LOCC group alone (represent scaffold group in our study).In contrary [29], reported that MSCs had no significant effect in sciatic regeneration compared to control group.

In proportion with [30], the scaffold group exhibited increased fibrous connective tissue content between muscle fibres and high collagen fibres compared with other treated groups. Mixed PRP and Adipose group showed the least collagen content compared to other treated groups. There were no statistical significance difference detected between both PRP and Adipose group [18]. indicated that gastrocnemius muscle fibres were more abundant in the LOCC/hUC-MSCs group than in the LOCC group (scaffold group) [7]. concluded that, nongrafted group has serious muscle atrophy, adipocyte hyperplasia, and many collagen fibres were seen in compared to autografted and TENGs groups.

Histopathologically, Schwan cell proliferation was highly pronounced in PRP + ADSCs group, despite of scaffold group which revealed a potent fibrous tissue proliferation instead of axonal growth in comparing to the contralateral normal nerve. The later result in line with [39] who explained that the distal portion of nerve sections in TENG group showed numerous regenerated nerve fibres with an even distribution in compared with non-grafted group.

Both ADSCs group and PRP group showed numerous regenerated fascicles with moderate axonal alignment were observed in the middle part of nerve conduit continued to the distal part with obvious Schwann cells proliferation and newly formed blood capillaries. This was in dispute with [29] who said that the absolute number of neural axons (number/µm2 ) distal to nerve repair was significantly higher in PRP group than the MSCs group. In agreement with [30], the distal nerve stump of grafted groups (ADSCs, PRP and ADSCs mixed with PRP) showed densely regeneration into the original fascicles with an even distribution in compared to nongrafted dogs that exhibit only obvious hyperplasia of connective tissues and disoriented arrangement of fusiform cells in degenerated fascicules. In addition [18], showed a more intense positive signal in the middle-portion of the nerve segment in the LOCC/hUC-MSCs group compared with the LOCC-alone group. Furthermore [6], said that bone marrow stem cell (BMSC) and autograft groups, massive bundles of myelinated nerve fibers, accompanied by numerous blood vessels, were observable at12 months post-surgery.

PRP was reported to exert its effect in the healing of the PNI via different mechanisms as; neuroprotection and averting the death of neurons, support axonal and vascular regeneration, control of the microenvironment’s inflammatory response, compensation of nerve-collateral muscular atroph**y** [13].

The part dissolved growth factors play in nerve regeneration is connected to the function of paracrine AdMSC (adipose mesenchymal stem cells). To aid in healing, these growth factors can shield tissue, increase vascularity, or reduce host inflammatory processes. AdMSC, under the direction of resident Schwann cells, were able to use host cells to facilitate intrinsic repair [40].

Remyelination observed in treated groups was happened by synthesis of neurotrophic factors like NGF from newly formed Schwann cells proliferated from mother cells used (adipose derived stem cells) or by the way through the effect of autologous injected PRP that enhance Schwann cell proliferation and migration [41]. Also, PRP is rich in many growth factors like VEGF “Vasculogenesis stimulation and increasing the perifollicular vessel size” and PDGF “Angiogenesis stimulation” and we determined their gene expression by a quantitative real-time PCR.

Nerve growth factor (NGF) is one of the neurotrophic factors secreted from active SCs after its proliferation and migration was triggered by PDGF-A. It is responsible for the formation of new nerve fibers in the Bunger band or tunnel tube for further proliferation and nerve regeneration from Wallerian degeneration to axonal remyelination. Its expression was up-regulated in proximal portion of all treated groups reflecting the axonal sprouting noticed in the proximal stump [1, 8] showed that adipose derived stem cells have the ability to secrete many growth factors among them was NGF whose expression was increased in treated group in compared to control group that was in a great establishment with our findings where PRP, ADSCs and PRP + ADSCs groups exhibit a significant change in NGF expression than scaffold group.

In a study evaluating the effect of PRP loaded nerve guidance conduit in recurrent laryngeal nerve injury; the expression of NGF in Schwann cells was increased in a dose-dependently. This implies that PRP may boost NGF secretion by activating SCs, and that PRP at higher doses may encourage SC growth [42].

The impact of ADSCs on NGF expression in Schwann cells following nerve damage has been the subject of numerous investigations. After injury, rats’ sciatic nerves were implanted with ADSCs which led to an increase in NGF expression in Schwann cells when compared to the injury-only group [43, 44]. In a different investigation, combining ADSCs and ANA graft transplantation showed functional recovery and nerve regeneration and promoted the repair of peripheral nerve injury over a 10 mm gap defect in rats which marked increase in neurotrophic factors including NGF over 12 months in the regenerated nerve tissue [8].

ADSCs that are injected into the damaged nerve produce neurotrophin-4, glial-derived neurotrophic factor, BDNF, and NGF to stop the loss of neurons in the dorsal root ganglia. While AdMSC can undergo neurogenic transformation, the majority of in vivo investigations have not shown that AdMSC implanted into neurons directly differentiate [40]. The ability of AdMSC to regenerate is currently believed to be influenced by paracrine factors than by the differentiation of AdMSC [44–48]. Numerous investigations have demonstrated that conditioned media derived from AdMSC culture has higher levels of several neurotrophic factors, including GDNF, NGF, and BDNF [38, 45, 49–51].

VEGF is one of the derivatives secreted via platelet degranulation and it is highly specific to vascular endothelium proliferation and migration through its chemotaxis effects so, it considered a critical modulator of angiogenesis during regeneration of peripheral nerves and promotes the neuronal survival and axonal growth [52, 53]. The expression of VEGF gene was highly up regulated in the proximal part of PRP + Adipose group by 3.7 fold which reflected in the evident revascularization picture observed by histopathological analysis matched with [54] who investigate the effect of VEGF-A as a neurotrophic factor for nerve recovery in rats and he found that a higher levels of VEGF-A were observed 2 weeks after nerve decompression and remained elevated after 4 weeks (*P* < 0.001) by using Western Blotting technique.

In a study evaluating the effect of PRP on axon development in spinal cord tissue, neutralizing antibodies against VEGF were added to the cocultures with PRP. The findings showed that adding PRP to the cocultures accelerated the growth of the axons, and adding neutralizing antibodies against VEGF dramatically inhibited the growth of the axons [55] [56]. demonstrated that injection PRP into sciatic nerve crush injury rabbit model; resulted in increased the expression of the VEGF in the injured nerve over 12 weeks post operation with enhanced axonal regeneration and recovery.

VEGF-A and VEGF165b, derived from AdMSC and AdMSC-CM, are effective at reducing pain levels in oxaliplatin-treated neuropathic mice [57]. Given that PRP stimulates angiogenesis and endothelial cell proliferation, it is thought to be a promising strategy to expand the uses of **ASCs** [58, 59]. Studies conducted both in vivo and in vitro have demonstrated that PRP and ASCs work better together to retain fat volume than they do separately. PRP was discovered to contribute to the enhancement of nerve regeneration in a rat sciatic crush injury model [58].

Also, Schwan cell proliferation and migration from the nerve stump is greatly affected by cytokines secreted from PRP and among them PDGF-A which considered the major influencer on SCs biological behavior. Pereira et al. [60] demonstrated that a human SCs cultured invitro with a low concentration of P-PRP were mainly enhanced by PDGF antibodies secreted from platelet and these antibodies are positively counteracted SCs proliferation and differentiation into myelin sheath. Gene expression of PDGF-A was markedly pronounced in the distal portion of PRP + Adipose group whose axonal alignment was highly organized and mannered in compared to other groups and this evidence were in the same way with [60] who proved that a VEGF-treated mice showed better functional performance after a sciatic nerve injury. Furthermore, MSCs produce angiogenic factors such as VEGF and PDGF [61].

Regarding PDGF, studies have demonstrated that neurons express PDGF receptors, and that PDGF-β is a mitogen and survival factor for Schwann cells on neurons [62] that exhibit trophic activity. Furthermore, following peripheral nerve damage, increased PDGF-β expression in peripheral neurons has been observed, indicating a potential function for PDGF-β in peripheral nerve regeneration [21]. According to a different study, PDGF enhanced nervous system regeneration and remyelination [63].

## Conclusion

In the current study, Group IV (PRP + ADSCs) showed the highest potential for sciatic nerve regeneration over ADSCs and PRP group through histopathological findings of increased Schwan cell and axonal fibers proliferation and up-regulation of NGF in the proximal and distal portion of nerve segment, also PDGF-A, VEGF in the proximal segment. Future research should therefore take this circumstance into account. before the recommendation for future application in clinic for any sciatic nerve affections. The present study has several limitations that warrant consideration; the gap created is 40-mm, but the maximum gap and appropriate timing of implantation after injury were not evaluated. Also, the effectiveness of the different treatments (ADSCs, PRP, and PRP + ADSCs) was investigated on the nerve transcriptome level without regarding the proteomic level. Hence, further long term studies with larger clinical samples size are required to confirm our findings and conclusion.

**Fig. 1:** Showed the application of neural tube between the two nerve stumps. (**A**) Illustrate suturing the neural tube with the proximal nerve stump using vicryl 4.0 suture. (**B**) Illustrate the application of injected therapy (PRP and PRP + ADSCs on sodium alginate) using a sterile nozzled syringe until filling the entire lumen of the tube (about 40 mm long). (**C**) Illustrate the length of the applicated tube after sutured with distal nerve stump filling the sciatic nerve gap

**Fig. 2:** Showed induction of sciatic nerve injury in dog, (**A**) Right thigh region, (**B**) Exposed sciatic nerve (**C**) Cutting of 2 cm of sciatic nerve, and (**D**) Sciatic nerve cut

**Fig. 3:** Demonstrates flow cytometric result and differentiation power of ADSCs. (**A**) Illustrate Flow cytometric analysis of ADSCs third passage. Cells were positive for CD73 (96.04%), CD105 (92.04%), CD9 (90.04%) and CD44 (88.02%) while negative for CD34 (0.16%) and CD45 (0.56%) while (**B**) show the differentiation capacity of ADSCs on adipogenic, osteogenic and chondrogenic media. Safranin O (**A**), Oil Red O (**B**) and Alizarin Red S (**C**) showed positive staining reaction with ADSCs.

**Fig. 4:** Illustrates significant difference of lameness score between different treated groups where ADSCs and PRP groups showed the highest score in compared to scaffold and PRP + ADSCs groups

**Fig. 5:** Showed the different electrophysiological parameters measured for all treated groups after one and six months from surgery: scaffold group showed marked reduction in the amplitude of compound muscle action potentials after 6 months in compared to other groups whereas adipose and PRP + ADSCs groups showed significant increase in the amplitude and significant reduction in the ratio of degeneration after 6 months in compared to first month (*P* ≤ 0.0001) values are presented as mean ± SD where *n* = 3/ group

**Fig. 6:** Photomicrograph illustrating the morphological analysis of the regenerative sciatic nerve in proximal, middle, and distal parts at different experimental groups (H&E): Red head arrow indicate: Schwan cells proliferation, black head arrow: indicate fibrous tissue, black arrow indicates demyelination and digestion chamber and red arrow indicate well developed blood vessels. scale bar : 50 μm

**Fig. 7:** Histochemical analysis of peripheral nerve regeneration and myelination. Figures showing the peripheral nerve regeneration pattern, degree of myelination (blue histochemical reaction) and collagen reorganization (red) with MCOLL histochemical in different experimental groups. Scale bar :15 μm

**Fig. 8:** Photomicrograph illustrating cross-sectional area of gastrocnemius muscle fiber (H&E) and collagen fiber content (MTC): Cross section of negative control group, Scaffold group showing marked muscular atrophy, hyperplasia of adipocyte (black head arrow) in addition to degeneration, necrosis, and hyalinization of muscle fibers (red head arrow) with stromal scirrhous reaction (red arrow), marked improvement in muscle diameter in PRP, ADSCs and PRP + ADSCS-groups. Collagen content with MTC stain (appeared blue in color) showing increase of collagen content in scaffold group, collagen content significantly reduced in the treated groups (PRP, ADSCs, PRP + ADSCs groups). scale bar :100 μm. Charts representing the cross-sectional area of gastrocnemius muscle fiber and area % of collagen fiber in different experimental groups. Values are expressed as means ± SD where *n* = 3/ group. Statistical analysis was performed using one-way ANOVA followed by Tukey’s multiple comparisons test. (*) indicates significance difference at *P* ≤ 0.05, (**) indicate significance difference at *P* ≤ 0.01, (***) indicate significance difference at *P* ≤ 0.001, (****) indicate significance difference at *P* ≤ 0.0001 (ns) indicate no significance

**Fig. 9:** The effect of different treatments for sciatic nerve after 6 months on the relative expression level of: (**A**) qRT-PCR results of nerve growth factor (NGF) gene for proximal nerve cut. (**B**) qRT-PCR results of nerve growth factor (NGF) gene for distal nerve cut. (**C**) qRT-PCR results of platelet derived growth factor-A (PDGF-A) gene for proximal nerve cut. (**D**) qRT-PCR results of platelet derived growth factor-A (PDGF-A) gene for distal nerve cut. (**E**) qRT-PCR results of vascular endothelial growth factor (VEGF) gene for proximal nerve cut. (**F**) qRT-PCR results of vascular endothelial growth factor (VEGF) gene for distal nerve cut Data were expressed as means ± SD (*n* = 3). (*) indicate significance difference at *P* ≤ 0.01, (***) indicate significance difference at *P* ≤ 0.001, (****) indicate significance difference at *P* ≤ 0.0001, (ns) indicate no significance

## Data Availability

Not applicable.

## Abbreviations

ADSCs: Adipose tissue-derived stem cells
CAMP: Compound muscle action potential
MCV: Motor nerve velocity
MSCs: Mesenchymal stem cells
NCV: Nerve conduction velocity
NGF: Nerve growth factor
PGA: Polyglycolic acid polymer
PRP: Platelet rich plasma
SCs: Schwann cells
TENG: Tissue engineered nerve grafts
VEGF: Vascular endothelial growth factor
